The article "Characterization and calibration of multiple 2D laser scanners" was published in 2022. Journal: PLoS One.

# Characterization and calibration of multiple 2D laser scanners

**DOI:** 10.1371/journal.pone.0272063

**Published:** 2022-07-28

**Authors:** Syed Riaz un Nabi Jafri, Sheraz Shamim, Sadia Muniza Faraz, Asif Ahmed, Syed Muhammad Yasir, Jamshed Iqbal

**Affiliations:** 1 Department of Electronic Engineering, NED University of Engineering and Technology, Karachi, Pakistan; 2 Department of Computer Science and Technology, Faculty of Science and Engineering, University of Hull, Hull, United Kingdom; Al Mansour University College-Baghdad-Iraq, IRAQ

## Abstract

This paper presents the comparative evaluation of multiple compact and lightweight 2D laser scanners for their possible backpack based scanning and mapping applications. These scanners include Hokuyo URG-04LX, Slamtec RPLidar A1-M8 and Hokuyo UTM-30LX-EW scanners. Since the technical datasheets provide general information and limited working details, this research presents a thorough study on the performance of each scanner related explicitly to indoor mapping operations. A series of scanning experiments have been performed for the characterization of each scanner using statistical analysis. During the testing, all the scanning data has been recorded using Robot Operating System (ROS) and then computed in offline processing. In initial tests, each scanner’s drift effect on range measurements has been tested and presented in the relevant section of the paper. In continuation, the effect of various scanning distances on measurement accuracy has been evaluated and discussed. Later the impact of various materials typically found in indoor vicinities and their respective properties of color and smoothness have been tested and provided in the paper. Finally, a Kalman Filtering based mathematical formulation has been utilized to calibrate each scanner and to reduce the measuring uncertainties as observed in various tests for each scanner.

## 1. Introduction

The laser scanners are extensively used in domestic and industrial automation applications for environmental sensing and providing accurate range-bearing information of surrounding objects. These scanners can be utilized on stationary platforms to detect moving objects such as products passing on the conveyer belt systems. On the other hand, they can be mounted on moving objects such as rovers to detect stationary and other moving objects passing around. In each scenario, polar range-bearing scan points of the surrounding objects, present randomly at specific orientations, are the most essential information which can be gathered through scanners. Using the perceived scan information, the shape of the object and its corresponding details can be extracted through multiple algorithms. With the advancement in the sensor’s manufacturing technologies, different 2D and 3D laser scanners are available for industrial, medical and agricultural applications [1].

Several past research works have reviewed the applications and advantages of 3D laser scanning in construction industry [2]. Many researchers have focused on working on 3D range information perceived through compact 3D laser scanners such as Velodyne lidar [3]. Multiple articles related to different 3D scanning products for indoor mapping applications have been published in recent years, providing performance evaluations of these products. The information related to mechanical, electrical and functional specifications such as physical appearance, weight, sensor type, operating time and usage in different lighting conditions are also reported. A detailed classification of 3D laser scanning technology for the possible selection of suitable products according to various applications, such as Advanced Driver Assistance System (ADAS) are also reported [4]. A research group has examined the measurement procedures of Velodyne VLP-16 and presented its characterization results [5]. The warm-up effects, stability and range errors during the testing of the scanner have carefully observed. A 3D scanner from Robosense has been evaluated for characterization from the perspective of 3D environmental range measurements [6]. Some researchers have analyzed and compared the characteristics of two well-known scanners, SICK MRS 1000 and Velodyne VLP-16 [7]. A careful investigation has been carried out to compare warm-up times, range and axial errors. Recent advancements in new solid-state technology have brought innovations in the development of laser scanners by eliminating many moving parts to provide stable and accurate scans. Researchers have studied the characteristics of these laser scanning devices and presented their results related to drift, range errors, the impact of material and ambient conditions [8].

Further, these scanners have been tested for real-world applications for the autonomous ground vehicle (AGV) for object detection and safety. However, the cost of the 3D scanning system and the computational complexity restrict their applications in many domains. For different surveillance and autonomous applications, multiple rovers with precise position control and actuation system, are using low cost laser scanners for self-localization and map building tasks in order to safely navigate in the targeted terrains [9]. A recent survey on 2D laser scanning technology has discussed its application for building 3D maps of the surveyed regions [10]. The low cost 2D scanning solution has been analyzed and compared with the commercial 3D laser scanning system by scanning the region through various orientations to perceive the complete vicinity. The characterization and calibration results of the 2D laser scanner UST-20LX have reported in the research work [11]. A group of researchers presented model based simulations with 2D Hokuyo URG-04LX scanner [12]. They studied surface-light interactions and simulated measurement processes to estimate model parameters from real sensor measurements. Numerous studies have reported performance evaluation of specific scanners [13]. These studies of laser scanners are necessary to realize their working limits in specific applications and provide essential knowledge in addition to the given information available in their datasheets. Unique characteristics results have been narrated by researchers using 2D laser scanners installed on moving platforms [14]. Obstacle detection and collision avoidance techniques are also reviewed for such moving systems using low cost 2D laser scanners. There are various factors on which the scanners have been tested such as the performance at variable ranges and the drift in range values with the passage of time. These scanners play a vital role in localization, mapping and object detection tasks for lifelong navigational operations which demand a careful and thorough study of their behavior. Due to these requirements, different scanners have been evaluated rigorously to make them an essential part of rover systems. A compact UBG-04LX scanner has been examined and evaluated for mapping tasks by a group of researchers [15]. Due to its lightweight and simple interface, the scanner can be mounted easily on a moving or stationary system and as per demonstrated results, its performance has been found quite stable.

In contrast to rover based applications, the backpack scanning systems are very popular to establish a 3D map of the surveyed territory using an integration of multiple 2D laser scanners on such scanning systems [16]. In these approaches, researchers have utilized various laser scanners mounted on different orientations to perceive the environment from unique perspectives. In order to achieve the best performance of these systems, a meaningful analysis of multiple laser scanners is required. Researchers have presented a study to investigate the available scanning mechanisms of various laser scanners present in the market and revealed that electromechanical 2D laser scanners are the most precise and widely used sensors for taking measurements from any kind of moveable system [17]. Globally many companies are manufacturing such 2D laser scanners with various working properties specifically related to range, field of view (FOV) and scanning time. Moreover, in parallel to these properties, mechanical and electronic interfacing along with the cost of the scanners are the crucial factors to consider in order to select the appropriate unit. This research work is presenting a thorough study on performance evaluation and characterization of popular low cost and compact 2D laser scanners suited for indoor 3D surveying applications using backpack laser scanning systems. The scanners used in this work are Hokuyo URG-04LX, Hokuyo UTM-30LX-EW and Slamtec RPLidar A1-M8. They have significant variations in working properties and are highly applicable for providing solutions related to indoor mapping problems. In this study, various properties of these scanners are examined and evaluated by experiments conducted in indoor environments and results are discussed. Section 2 is presenting a summary of relevant research works. Section 3 is describing the specifications of selected scanners along with the details of the testing setup. Section 4 is providing the characterization of all scanners with respect to desired technical aspects. Section 5 is introducing the calibration model for the scanner followed by conclusions of the research work.

## 2. Related work

The performance evaluation and characterization of multiple 2D laser scanners have been performed by many researchers. In these research works, different technical parameters of these scanners that could affect their performances have been studied. Although available data sheets of these scanners provide knowledge of some technical aspects but they cannot entirely explain the working behavior of such scanners in particular applications. Designers of scanning systems need to know carefully about specific technical aspects such as the warm-up period, range errors in different lighting conditions, performance of the scanner for various target surface materials and scanner’s placement effect at different orientations.

A comprehensive research study on the performance of Time of Flight (ToF) based 2D and 3D laser scanners have presented by the authors and they provided eight qualitative and quantitative test procedures for examining the various behaviors of these scanners [18]. The scanners have testified for determining the warm-up time to identify temperature effects, impact on range and angular stepping accuracy, effects of ambient light, material variations, vibration and shock effects on scanning quality. A group of researchers presented a detailed characterization of the Hokuyo URG-04LX scanner [19]. They analyzed the scanning quality by varying the targeted surface properties such as material and color. They investigated the behavior of scanner under different lighting conditions on various surfaces. They also observed the generated range errors by varying the incidence angle due to changes in the scanner’s orientation and placement. A thesis study has investigated the application of a 2D laser scanner with a reflective superstructure to form a 3D perspective for airborne applications where weight is the primary concern for safe system operation [20]. In addition, the author introduced the calibration strategy for entirely scanning the surveying vicinity with acceptable accuracy. Some researchers have evaluated the performance of the 2D Hokuyo UST-20LX laser scanner for indoor operations and presented its characterization results for range error effects due to varying surface material properties and beam divergence [21]. Authors of research work have studied the performance of the 2D Sick LMS-200 scanner and compared it with the Hokuyo URG-04LX scanner [22]. They investigated the working capabilities of both scanners on different surfaces of complex shapes and analyzed their capability of accurately mapping the targeted object. Selection of appropriate scanners for suitable applications require a comparison of specific characteristics of both scanners with added advantages of cost-effectiveness, compactness, lightweight and lower power solution. The URG-04LX is a short-range and compact scanner with a compromising performance if compared with the presented results of the LMS-200 scanner. Therefore, the selection decision may vary as per the scanning system requirements and the designer can pick that scanner that fulfils maximum specific technical requirements. Another study has presented the working capabilities of the Hokuyo PBS-03JN scanner for indoor mapping applications [23]. Moreover, the study has compared PBS-03JN with LMS-200 and presented the relevant indoor testing results. Some authors examined the performance of the Sick LMS511-20100 Pro laser range finder for object detection and simultaneous localization and mapping applications [24]. They investigated its characteristics such as drift effect, range error, angular resolution, impact of target materials and provided guidelines for its optimal use.

The compact 2D laser scanners can be used for 3D mapping applications by integrating them at certain orientations. A group of researchers studied the performance of 2D scanners for 3D tasks and presented their evaluated results [25]. The calibration procedure described in this work provided an estimation of the internal parameters of the laser scanner for more accurate results. Similarly, the 3D mapping result has been investigated by researchers using the compact 2D laser scanner [26]. Another article presented characteristics and application results of the URG-04LX scanner for navigation estimation of walking robots [27]. In contrast to low range scanners, the Hokuyo UTM-30LX is another popular scanning product that has an extended scanning range of 30 m. This scanner has been used in many applications such as researchers have utilized it for the detection of obstacles along the overhead power lines using the moving robot [28]. Due to its compactness and lightweight, many mobile robots have been integrated with this scanner and detailed characterization results for mapping and object detection applications have presented in a research work [29]. A group of researchers have performed a comparison of UTM-30LX with a multi-layer IBEO LD-ML scanner and presented measurement characteristics during rain, dust and other environmental conditions [30]. Multiple probabilistic models have been tested for the same UTM-30LX scanner by other researchers and proposed a pre-processed range data fusion technique to improve the scanning error of the unit [31].

Some new low range and economical 2D laser scanner units have emerged in the past couple of years such as the RPLIDAR A1 scanner unit. This scanner is compact, low power and easy to interface however it is more sensitive to sunlight. The scanner has been utilized in many research works for mobile robot navigation and mapping applications. An algorithm has been proposed for the localization of multi-robots in an indoor environment using RPLIDAR scanners integrated on each rover [32]. A research group has utilized the scanner for 3D indoor mapping application in absence of the room light and presented satisfactory results with respect to ground truth [33]. In general, all 2D laser scanners utilized by researchers have some definite useful properties along with some technical and financial drawbacks. The scanners that have been considered and examined in this research study are cost effective and compact scanners that can interface with backpack scanning systems for indoor mapping applications. In the next sections of this paper, a comparative analysis of various scanners is presented and experimental testing results are explained for the understanding of technical properties of such scanners.

## 3. Comparison of multiple 2d laser scanners

There are various 2D laser scanners designed to operate in numerous environments and provide the benefit of non-contact sensing of the surveyed region. Based on general features of scanners such as compactness, interfacing and cost, three 2D laser scanners including Hokuyo URG-04LX, Hokuyo UTM-30LX-EW and RPLidar A1-M8, have been selected to examine their characteristics specifically for backpack based indoor surveying operations. The manufacturers provide the general technical specifications of the respective scanner in order to verify the application suitable for the relevant scanner. This section is presenting the comparison and general performance evaluation based on the provided information available in the datasheets of these scanners.

### 3.1. Performance evaluation of multiple 2D laser scanners

The selected three 2D laser scanners under evaluation have been shown in Fig 1. Hokuyo laser scanner series provides a compact and multiple ranges of scanners for cost effective solutions related to self-localization and mapping tasks. A popular low range 2D laser scanner is Hokuyo URG-04LX which is quite a compact and accurate scanner [34]. It can scan a planar area around the scanner within 4 m of range having a scanning angle span of 240◦ and can deliver scans with a frequency of 10 Hz. Its technical parameters have been summarized in Table 1. A recently developed series of scanners is RPLidar which are producing compact low range scanners at affordable costs. One of the pioneer scanners from this series is RPLidar A1-M8 2D laser scanner as shown in the middle of Fig 1 [35]. It can completely scan a planar area around it within 6 m of range with a 360◦ angular view and can deliver scans with a frequency of 5.5 Hz. It is comparatively less accurate and delivers a compromised performance at a highly affordable cost. Its technical specifications have been provided in Table 1.

**Fig 1:** 2D Laser scanners (left) URG-04LX (middle) RPLidar A1 (right) UTM-30LX.

**Table 1:** Specification of 2D laser scanners.

Parameter	URG-04LX	RPLIDAR A1-M8	UTM-30LX
Maximum measurement range (m)	4	6	30
Measurement error (mm)	±10mm up to 1m range; 1% of measurement value for 1-4m range	±50	±30mm for 0.1 to 10m range, ±50mm for 10 to 30m range
Scanning angle (deg.)	240	360	270
Angular resolution (deg.)	0.36	≤ 1	0.25
Scanning time (ms/cycle)	100	180	25
Measurement resolution (mm)	1	< 0.5	0.1
Data interface and transfer rate	RS232, USB 2.0	USB 2.0	USB 2.0, Ethernet port
Supply voltage (VDC)	5± 5%	5± 5%	12±10%
Current consumption (mA)	500	350	700
Weight (kg)	0.16	0.2	0.37
External dimensions (WxLxH in mm)	50 × 50 × 70	90 × 70 × 60	62 × 62 × 87.5
Cost($)	2000	400	7000

Another Hokuyo medium range scanner UTM-30LX is selected as shown on the right side of Fig 1 [36]. It is capable to scan with an increased range of 30 m with a scanning angle span of 270° at a scanning frequency of 40 Hz. This scanner is highly accurate and robust but expensive. Its technical specifications have been shown in Table 1.

The specifications provided by the manufacturers as summarized in Table 1 highlighted the basic performance and behavior of such scanners and cannot cover the detailed comparative performance in any specific application. The impact of properties of targeted objects such as material, color and smoothness can influence the performance of the scanner. Moreover, the longer usage of scanners may cause the drift in range measurements which needs to identify. Therefore, a planned investigation is needed to study the performance and characteristics of each scanner in the actual environments as presented in the next section. The analysis of characteristics helps the designer of the scanning system to predict the possible inaccuracy of measurements and to minimize its impact on the system performance.

### 3.2. Experimental setup

In order to evaluate the characteristics of different scanners, an experimental multi-floor scanner’s mounting platform has been designed in SolidWorks CAD software as shown on the left side of Fig 2. The mechanical CAD model has been designed in such a manner that on each floor, a single scanner can be placed and its central position has been set concentric to the remaining scanners. After completing the CAD design, the real manufacturing of the platform has been performed. The Aluminum metal sheet of thickness 5 mm has been selected due to its strength, durability and lightweight characteristics to make each floor of 155 mm x 155 mm dimension. All three squared floors have been assembled with the help of thin aluminum pillars of 115 mm height to provide sufficient place for fixing each scanner. Later all three scanners have been mounted horizontally as shown on right side of Fig 2. The UTM-30LX has been assembled at the bottom, URG-04LX and RPLidar A1 have been placed at the middle and top floor plates respectively. Since only RPLidar A1 can perform a 360° full scan so it has been mounted on the top floor to avoid any obstruction in range measurement. During testing, it was critical to keep scanners in uniform position with a clear scan vision for reliable data recording. It has been achieved through the manufactured platform.

**Fig 2:** Experimental setup (left) 3D CAD model (right) real hardware.

The instrumentation scheme of the experimental setup has been shown in Fig 3. All three scanners have been interfaced using USB ports to the Robot Operating System (ROS) which was installed on the laptop [37]. ROS has the ability to initialize and interface multiple sensors including these three scanners. Moreover, online data logging and storage can be done to do offline processing. In all experiments conducted in this research work, online data recordings have been performed for all scanners and later the recorded scan data files have been visualized and processed using Matlab scripting as shown in Fig 3. The time synchronization and outlier rejection have been performed from each scan file. Later, computational analysis has been performed to determine statistical parameters of mean, standard deviation and root mean square error (RMSE) on samples of scans recorded in different experiments. Finally, calibration modeling has performed on each scanner.

**Fig 3:** Instrumentation system design.

## 4. Characteristics of laser scanners in indoor environment

The scanner’s platform has been placed inside an indoor lab as shown on the left side in Fig 4 in order to study the characteristics of each scanner. The interior of the indoor lab has been set up specifically to hold common furniture items, which may present in various indoor environments while conducting scanning jobs using the backpack system. In general, the lab structure is consisting of concrete walls and pillars, a tiled floor, a false ceiling, wood doors and windows. The lab furniture is comprised of wooden tables, steel cabinets and plastic objects. The scanning platform has been placed at an end of the lab in such a way that the majority of the furniture has appeared in front of the platform which can be viewed by the individual scanner as indicated by a scale less sketch of the lab on the right hand side of Fig 4. The reference frame of the platform has been shown by red arrows labeled as X_P_ and Y_P_ for the XY axis and it has served as the origin of all scan measurements. Depending on the range specifications of each scanner, respective furniture items have been perceived in the individual scans. Multiple tests have been conducted with different time intervals for observing drift effect, range variations and influence of the target’s properties such as the color and material of the object.

**Fig 4:** Indoor experimental setup (left) Lab environment (right) Conceptual picture.

The first test has conducted in the indoor lab and a sample of the range scan of URG-04LX has shown in Fig 5. The scanner has perceived those objects which are in its four-meter range within a 240° field of view. Many surrounding objects including concrete walls, vinyl sheet, steel cabinet and some tables have been detected by the scanner and their respective scan points have been shown in red color. The partial structure of walls has been scanned due to the presence of objects in between the scanner and walls. Some objects such as Table 2 have been scanned completely as shown in the figure and its central scan point has been marked by a red circle however deviations due to the scanner’s noises in other range points are visible.

**Fig 5:** Laser scans of indoor environment of URG-04LX.

**Table 2:** Comparison of drift effects of 2D laser scanners at four meter distance.

Scanner	Mean Value	Standard Deviation	Relative Error	RMSE
	${\overset{-}{x}}_{M}\;$(mm)	${\overset{-}{\sigma }}_{M}$ (mm)	${\overset{-}{\eta }}_{M}$ (%)	(mm)
URG-04LX	3986.3	16.8	-0.34	14.35
RPLidar A1	4017.3	21.3	0.43	17.2
UTM-30LX	4006.6	11.3	0.16	6.3

A sample of the range scan of RPLidar A1 has shown in Fig 6, which perceived those objects present within a six meter range of around 360°. The origin of the scanner has shown by a red reference frame labeled by X_P_ and Y_P_. Multiple surrounding objects such as wall 1 and Table 2 can be viewed by green scan points in the figure with visible deviations among them.

**Fig 6:** Laser scans of indoor environment of RPLidar A1.

Similarly, the sample range scan of UTM-30LX has been presented in Fig 7 and it is showing scanned objects present within the 14 m range inside a 270° field of view. This scanner has a greater scanning range of thirty meters but the application region has dimensional limits therefore only already placed objects have been analyzed in its scan. Many surrounding objects such as wall 1 and multiple tables can be viewed by blue scan points in the figure with visible deviations among them.

**Fig 7:** Laser scans of indoor environment of UTM-30LX.

The experimental data for multiple tests have been recorded for certain time durations as required and computed offline to evaluate the statistical results of each scanner. The overall procedure has been presented in the flow chart as shown in Fig 8.

**Fig 8:** Flow chart of overall testing procedure.

As, pointed in the flow chart, due to high frequency of incoming scans, some samples at regular small intervals have been selected and processed from the overall population of scans. In order to evaluate the scanning stability, any particular object such as Table 2 has been selected and its central location as marked by the red point in Fig 5 has been observed for the ongoing scanning test. Let’s say its specific range value for *i*^th^ sample scan of a respective scanner is *x*_*i*_ and there are *N* no. of sample scans have recorded in a certain *m*^th^ time interval of one minute so the sampled range mean value ${\overset{-}{x}}_{m}$ for the red middle point can be determined using Eq (1).


$${\overset{-}{x}}_{m}=\frac{1}{N}\sum_{i=1}^{N}x_{i}$$ (1)

The sampled standard deviation *σ*_*m*_ at *m*^th^ time interval is calculated by using Eq (2).


$$\sigma_{m}=\sqrt{\frac{1}{N}\sum_{i=1}^{N}(x_{i}-{\overset{-}{x}}_{m}{)}^{2}}$$ (2)

The signed error term *e*_*m*_ for this time interval is calculated by computing the difference between the true value *x*_*T*_ and the measured mean value ${\overset{-}{x}}_{m}$ as shown in Eq (3).


$$e_{m}=x_{T}-{\overset{-}{x}}_{m}$$ (3)

The percent relative error *η*_*m*_ is computed using the error term and true value as shown in Eq 4.


$$\eta_{m}=\frac{e_{m}}{x_{T}}\times 100$$ (4)

The above calculations have been performed for the complete duration of the test for *M* regular time intervals and overall single average values for mean ${\overset{-}{x}}_{M}$, standard deviation ${\overset{-}{\sigma }}_{M}$ and relative error ${\overset{-}{\eta }}_{M}$ for whole the test using individual values have computed as shown in Eqs (5)–(7).


$${\overset{-}{x}}_{M}=\frac{1}{M}\sum_{m=1}^{M}x_{m}$$ (5)

$${\overset{-}{\sigma }}_{M}=\frac{1}{M}\sum_{m=1}^{M}\sigma_{m}$$ (6)

$${\overset{-}{\eta }}_{M}=\frac{1}{M}\sum_{m=1}^{M}\eta_{m}$$ (7)

Furthermore, the root mean square error (RMSE) for complete test duration has computed using all *M* number of error terms as shown in Eq (8).


$$RMSE={\left[\frac{1}{M}(\sum_{m=1}^{M}e_{m}^{2})\right]}^{1/2}$$ (8)

After analyzing the response of range values belonging to Table 2 of all scanners, another object such as Table 3 has been selected which has different range measurements from all scanners. It has also been examined to see the respective scanner’s response. The following sections are presenting the required analysis and related discussions using the described procedure.

**Table 3:** Comparison of drift effects.

Scanner	Target Distance	Mean Value	Relative Error
	(mm)	${\overset{-}{x}}_{M}\;$(mm)	${\overset{-}{\eta }}_{M}$ (%)
URG-04LX [19]	1500	1475	-1.6
URG-04LX [22]	3600	3625	0.7
UTM-30LX [28]	1000	1002	0.2
UTM-30LX [29]	2000	2030	1.5
UTM-30LX [30]	2000	2012	0.6

### 4.1. Drift effect

Normally laser scanners exhibit drift in range values even for stationary objects due to the warming effect generated inside their structures. It may occur due to the heat dissipations of the spindle motor and the electronic circuitry itself, which result in a continuous increase of the operating temperature of the scanner. It is considered as a very important characteristic of any laser scanner and is needed to identify the influence of the warming of a scanner on measured range values over a specified period. In order to understand the drift effect, an experiment has conducted in the indoor lab at normal room temperature and lighting conditions. Before the test, each scanner was in off condition for more than twelve hours. The test has conducted for more than thirty minutes to record the warming effects of each scanner. This duration has been selected because the available backpack scanning system has a battery power limit of forty minutes therefore the performance of each scanner needs to evaluate within this working time. Multiple target objects have been placed at variable distances as explained earlier in Fig 4. One of the wooden table placed at four meters at an incidence angle of nearly five degrees has been selected and its scan observations of the middle point from each scanner has recorded and evaluated. The range plots *x*_*i*_ of sampled scans of URG-04LX has shown in blue color in Fig 9. The sampled mean values ${\overset{-}{x}}_{m}$ have been plotted in green color in the same figure. The few outlier measurements if detected have not been taken into consideration. The blue range and green mean plots are indicating a slow shift in values with the passage of time and acquire comparatively stable working approximately after fifteen minutes. This behavior has been observed in some other tests and it is evaluated that the range drifts of URG-04LX have reached stability after fifteen to twenty minutes of operation. Therefore a safe backpack scanning system may initiate after twenty minutes of energizing the scanner and can last for twenty minutes with the available capacity of energy source. The overall mean ${\overset{-}{x}}_{M}$, standard deviation ${\overset{-}{\sigma }}_{M}$, relative error ${\overset{-}{\eta }}_{M}$ and RMSE values of the complete test have shown in Table 2.

**Fig 9:** Drift test of URG-04LX using range measurements of four meter distance.

The range drift behavior of the RPLidar scanner has been observed on the same table object. The range plots *x*_*i*_ of sampled scans of RPLidar has shown in blue color in Fig 10. The sampled mean values ${\overset{-}{x}}_{m}$ have been plotted in green color in the same figure. The blue range and green mean plots are indicating a continuous slow shift in values with the passage of time till the end of the experiment. Some other tests have also indicated almost the same responses which means that the RPLidar scanner has not reached to range stability within a given time duration and may produce small range errors for those scanning systems where power limits exist. This behavior may be due to the usage of low-cost components and scanner casing as this system has been produced for very economical applications. Respective mean and standard deviation values have been provided in Table 2.

**Fig 10:** Drift test of RPLidar using range measurements of four-meter distance.

Finally, the UTM-30LX scanner has been tested and its drift effect has been evaluated on the same table. The range plots *x*_*i*_ of sampled scans of UTM-30LX has shown in blue color in Fig 11. The sampled mean values ${\overset{-}{x}}_{m}$ have been plotted in green color in the same figure. The blue range and green mean plots are indicating very minute deviations in measured values with the passage of time. Some other tests have witnessed almost the same responses, which means that the UTM-30LX scanner has offered range stability quickly and its range values can use after few minutes of its energizing. This attractive behavior is due to the usage of better quality components and scanner casing however all great features have been offered at a higher cost. The overall statistical values of the test have been shown in Table 2 which is indicating the relatively better performance of the scanner as compared to other tested scanners.

**Fig 11:** Drift test of UTM-30LX using range measurements of four-meter distance.

Many research groups conducted drift test for URG-04LX and UTM-30LX with different time durations. The provided results are in agreement with results stated in Table 2. However, the relative error values for URG-04LX were found greater as summarized in Table 3 due to longer test duration as compared to their values stated in Table 2 [19, 20]. Similar observations have been found for the tests related to UTM-30LX and the relative error values were greater for long drift tests as highlighted in Table 3 [28, 29, 30].

### 4.2. Impact of target distance on range measurements

The scanning quality of any scanner in a respective environment depends on measuring range stability for dispersed objects present in the vicinity at various distances from the scanner. This section presents the responses of individual scanners for sensing distant objects and their effects on respective range measurements. This analysis is very important for understanding the level of accuracy of the specific scanner at various range measurements and the possibility of using it in map development applications. To understand the impact of range variations, three distinct table objects have been selected present in the indoor vicinity at different distances of nearly two, six and twelve meters from the scanning platform and have been scanned continuously for thirty minutes. Considering range measurements of the middle position of the second table object present at two point four meters, plots of the mean range values along with the standard deviations of URG-04LX have shown in Fig 12. Both parameters have visible variations in the beginning but after fifteen minutes of operation, they reached almost constant values with minimum deviations.

**Fig 12:** Range plot of URG-04LX for measuring stability test for object present at 2.4m distance.

For the same table, the mean range and standard deviation plots of RPLidar have shown in Fig 13. Both values have depicted minute variations throughout the test and no stability has been reached.

**Fig 13:** Range plot of RPLidar for measuring stability test for object present at 2.4m distance.

The respective plots of both parameters related to UTM-30LX have shown in Fig 14 where these parameters have reached stability after fifteen minutes. Table 4 is presenting the respective statistical results of each scanner where UTM-30LX has indicated better performance. Overall performances of the other two scanners were found satisfactory indicating that low-cost scanners can be used with a compromised performance for short range applications.

**Fig 14:** Range plot of Hokuyo-30LX for measuring stability test for object present at 2.4m distance.

**Table 4:** Comparison of measuring stability of 2D laser scanners at 2.4 m distance.

Scanner	Mean Value	Standard Deviation	Relative Error	RMSE
	${\overset{-}{x}}_{M}\;$(mm)	${\overset{-}{\sigma }}_{M}$ (mm)	${\overset{-}{\eta }}_{M}$ (%)	(mm)
URG-04LX	2398.2	12.2	-0.08	2.14
RPLidar A1	2395.1	17.1	-0.20	5.49
UTM-30LX	2401.7	8.2	0.04	1.36

Considering range measurements of the fourth table presents nearly six meters, which is out of range to URG-04LX. Plots of the mean range values along with the standard deviations of RPLidar have shown in Fig 15 where the standard deviation has significantly increased. Both parameters have greater variations as compared to earlier short range responses for the second table and again no stability has been reached in measurements.

**Fig 15:** Range plot of RPLidar for measuring stability test for object present at 6m distance.

However, the respective plots of both parameters related to UTM-30LX have shown better stability after ten minutes of operation as shown in Fig 16.

**Fig 16:** Range plot of Hokuyo-30LX for measuring stability test for object present at 6m distance.

Another fifth table object placed distantly nearly at twelve meters has been scanned only by UTM-30LX as the other two scanners have no sensing range for this object. Again both parameters have plotted as shown in Fig 17 where these parameters have reached stability after approximately twenty minutes.

**Fig 17:** Range plot of Hokuyo-30LX for measuring stability test for object present at 12m distance.

The accuracy of UTM-30LX scanner has been found better along with its stability which has reached approximately in twenty minutes and it provides the possibility of sensing greater ranges. In addition, it provides a higher number of scanned points related to any particular object due to its lower angular resolution as compared to the other two scanners. The standard deviation for UTM-30LX remains persistent for all observed objects and is found at a maximum nearer to ±15 mm while the maximum standard deviation observed for URG-04LX was nearly ±20 mm, however, its sensing range is very low which limits its usage related to mapping applications. The RPLidar scanner has reflected a significant increase of the standard deviation from ±12mm to ±40mm as the target range is increased. It is also observed that the relative error of RPLidar is higher than both Hokuyo scanners.

The range errors have also been determined by various research authors for URG-04LX and UTM-30LX by placing the targeted object at variable distances. The provided test results have appeared very similar and are summarized in Table 5 as compared to the results presented in Table 4. Some variations can be seen in relative errors for URG-04LX when the target distance has increased [19, 22]. The same testing at a higher target distance has been carried out by multiple researchers for UTM-30LX [28, 38]. As the scanned object has been placed at a distant place, so greater relative errors have been observed as shown in Table 5. The possible cause of this impact is the relatively greater spreading of the laser beam at higher distances and observing a low intense reflection of the beam reception at the scanner’s end.

**Table 5:** Comparison of range measurements.

Scanner	Target Distance	Mean Value	Relative Error
	(mm)	${\overset{-}{x}}_{M}\;$(mm)	${\overset{-}{\eta }}_{M}$ (%)
URG-04LX [19]	1000	987	1.3
URG-04LX [22]	3600	3625	-0.7
UTM-30LX [28]	1500	1505	-0.3
UTM-30LX [38]	1200	1220	1.6

### 4.3. Effect of various materials on range stability

The scanning vicinity holds multiple kind of objects of different materials. The main objective of this section is to observe the responses of individual scanners on various materials present in office or lab kind of environments for developing an accurate scanning system. In this experiment, four different target materials have examined which were present at multiple orientations and distances from scanners. The common materials used in objects present inside targeted indoor vicinities are concrete, wood, steel and plastic. These materials were analyzed according to the degree of surface smoothness at normal room light conditions. The multiple objects of vinyl plastic sheet, steel cabinet, concrete walls and wooden tables have been tested present at certain ranges as already shown in Fig 4. All the scanners have been powered up at the same time and continued to operate for thirty minutes. After twenty five minutes of operations, all measurements of each scanner have been recorded in order to reduce the impact of drift effect for initial measurements. The statistical calculations have been performed on recorded scanning data and are provided in Table 6. The true range values of objects and statistical values of each scanner have been plotted as shown in Fig 18. The results are indicating that the reflectiveness of the material has created an impact on the measurement accuracy of each scanner. The measurements of matt finished concrete wall, wood table and steel cabinet have shown higher accuracy if observed by the corresponding *RMSE* values of each scanner. The measurements related to comparatively shiny vinyl plastic object has shown less accurate results for all scanners even though the object was placed nearer to scanners in order to minimize the range stability effect. The overall performance of UTM-30LX has been found superior to other scanners and the maximum standard deviation was under ±13 mm along with comparatively smaller *RMSE* values. On other hand, UTM-04LX has shown reasonably accurate performance and its maximum standard deviation was under ±18 mm along with small *RMSE* values. While RPLidar has shown a mixed response with higher inaccuracies as compared to the other two scanners and its standard deviation and *RMSE* values reached to larger values as shown in the following table. However, for economical scanning operations at compromised performance, the RPLidar has presented a reasonable performance and it depends on the user needs that how much accuracy is needed if compared with the budgeting of the scanning system.

**Fig 18:** Plot of mean and standard deviation of each scanner by scanning different targeted materials.

**Table 6:** Effect of materials on range measurements.

Material	Scanner	Mean Value	Standard Deviation	Relative Error	RMSE
		${\overset{-}{x}}_{M}\;$(mm)	${\overset{-}{\sigma }}_{M}$ (mm)	${\overset{-}{\eta }}_{M}$ (%)	(mm)
Wood (True value: 4m)	URG-04LX	3985.3	17.6	-0.38	16.1
	RPLidar A1	4020.3	22.4	0.44	21.6
	UTM-30LX	4005.6	13.2	0.13	5.8
Steel (True value: 1.95m)	URG-04LX	1932.6	9.8	-0.12	19.4
	RPLidar A1	1929.0	12.4	-0.15	22.45
	UTM-30LX	1942.3	8.6	-0.09	8.7
Plastic (True value: 1.85m)	URG-04LX	1798.7	13.6	-3.2	52.3
	RPLidar A1	1789.8	16.7	-4.4	61.9
	UTM-30LX	1810.9	9.6	-2.2	39.1
Wall (True value: 3.4m)	URG-04LX	3387.3	17.8	-0.54	13.2
	RPLidar A1	3374.1	21.6	-0.63	25.5
	UTM-30LX	3393.7	11.8	-0.51	6.7

The effect of materials has been presented by researchers for all three scanners in different articles. In general, the stated results are closed to those presented in Table 6. However, some variations have been observed in relative errors due to the presence of various materials at longer distances as shown in Table 7 for URG-04LX [19, 22]. The same phenomena have occurred for UTM-30LX and are presented in Table 7 [29, 38, 39]. In addition, the presented results for RPLidar are quite similar as determined in the presenting work however due to variations in testing ranges, the stated result of relative errors is little bit higher [39].

**Table 7:** Comparison of effect of materials on range measurements.

Material	Scanner	Target Distance	Mean Value	Relative Error
		(mm)	${\overset{-}{x}}_{M}$ (mm)	${\overset{-}{\eta }}_{M}$ (%)
Wood	URG-04LX [19]	1599	1487	0.86
	URG-04LX [22]	3600	3652.2	-1.45
	UTM-30LX [29]	1500	1495	0.3
Steel	URG-04LX [19]	1500	1515	-1
	URG-04LX [22]	3600	3643.3	-1.20
	RP Lidar [39]	2000	2149.5	-7.4
	UTM-30LX [29]	1500	1504.5	-0.3
	UTM-30LX [39]	2000	2020.4	-1.02
Plastic	UTM-30LX [29]	1500	1493	0.46
Wall	UTM-30LX [38]	1200	1220	1.6

### 4.4. Dependency on color variations

The indoor surveying environments contain multiple colored objects, which may impact scanning quality. In order to see color dependency, simple scanning tests have been conducted in the indoor lab by placing different colored objects around the scanning platform, as shown in Fig 19. The variations in target color have been created by pasting the card paper sheets of multiple colors on tables placed at a fixed distance of four meters from the scanning platform. The scanning test has been performed for thirty minutes. The last five minutes readings have been used to analyze variations in range measurements due to changes in target color.

**Fig 19:** Indoor experimental setup for color test, (left) Blue (middle) Red (right) Green colored objects.

The plot of the mean and standard deviations of all three scanners for a red color object scanning test has shown in Fig 20. The values are indicating a more accurate response of Hokuyu-30LX as compared to the other two scanners. All the calculated statistical values have been provided in Table 5 in the respective row of red color object. These measured values can be compared with the earlier test values provided in Table 2 where the same table object with its original brown color was scanned. Both test values are very closer and reflect almost the same responses for all scanners. All the values such as mean and *RMSE* of each scanner are looking identical and it is reflecting that no significant change has occurred by changing the color of the targeted object.

**Fig 20:** Plot of mean and standard deviations values for red color object.

The plot of the mean and standard deviations of all three scanners for a blue color object scanning test has shown in Fig 21. The Hokuyu-30LX has shown more accurate results however again no indication of a different behavior has been observed if compared to the statistical values observed as mentioned in Table 8 for the respective blue color. The other two scanners have an almost similar response, only a few units of *RMSE* of RPLidar has increased.

**Fig 21:** Plot of mean and standard deviations values for blue color object.

**Table 8:** Impact of color variations on range measurements.

Color	Scanner	Mean Value	Standard Deviation	Relative Error	RMSE
		${\overset{-}{x}}_{M}\;$(mm)	${\overset{-}{\sigma }}_{M}\;$(mm)	${\overset{-}{\eta }}_{M}\;$(%)	(mm)
Red	URG-04LX	3985.2	11.5	-0.35	16.2
	RPLidar A1	4019.3	15.4	0.58	19.6
	UTM-30LX	3995.6	7.8	-0.12	5.1
Blue	URG-04LX	3988.4	10.7	-0.31	13.6
	RPLidar A1	4029.1	12.4	0.77	27.4
	UTM-30LX	4006.7	6.3	0.15	7.3
White	URG-04LX	3992.1	12.3	-0.18	8.7
	RPLidar A1	4021.3	17.6	0.61	21.8
	UTM-30LX	3994.9	7.8	-0.13	5.2
Green	URG-04LX	3985.8	11.2	-0.35	15.1
	RPLidar A1	4023.1	14.8	0.63	23.4
	UTM-30LX	3999.2	8.7	-0.03	1.1

The plot of the mean and standard deviations of all three scanners for a white color object scanning test has shown in Fig 22. There are similar responses observed for all scanners and provided in the respective column of Table 5.

**Fig 22:** Plot of mean and standard deviations values for white color object.

The plot of the mean and standard deviations of all three scanners for a green color object scanning test has shown in Fig 23. All statistical values of all scanners have been provided in Table 8 and it concludes that no major variations have been observed in different parameters including mean and *RMSE*, only standard deviations have been a little bit varied in multiple tests by changing the target color if providing constant lighting conditions during all experiments.

**Fig 23:** Plot of mean and standard deviations values for green color object.

The scanning tests on various colored objects have been performed in a variety of research works. No significant observations have been reported due to the change of color. Some provided results for URG-04LX have been summarized in Table 9 [19, 22]. Similarly, the scanning results for UTM-30LX have listed in Table 9 for different research works and no unique observation has been observed as stated in related articles [28, 29, 40].

**Table 9:** Comparison of impact of color variations.

Color	Scanner	Target Distance	Mean Value	Relative Error
		(mm)	${\overset{-}{x}}_{M}$ (mm)	${\overset{-}{\eta }}_{M}$ (%)
Red	URG-04LX [19]	1500	1476	1.60
	URG-04LX [22]	3600	3648	-1.33
	UTM-30LX [29]	1500	1489	0.73
Black	URG-04LX [19]	1500	1485	1.00
	URG-04LX [22]	3600	3649	-1.36
	UTM-30LX [28]	1500	1504	-0.27
	UTM-30LX [29]	1500	1492	0.53
White	URG-04LX [19]	1500	1480	1.33
	URG-04LX [22]	3600	3649.9	-1.39
	UTM-30LX [29]	1500	1483	1.13
Green	URG-04LX [19]	1500	1470	2.00
	UTM-30LX [29]	1500	1489	0.73

## 5. Calibration of individual scanners using Kalman Filter

All the experiments conducted and presented in earlier sections are indicating that each scanner has reflected noises in respective range measurements. The magnitudes of the noises are obviously uncertain and can be changed in successive experiments as observed in Tables 2, 4, 6 and 8 from the values of mean and standard deviation, however, they were always found within the limits as listed in datasheets of the scanners and as summarized in Table 1. There are many popular mathematical implementations that have been provided to minimize noises and uncertainties in range measurements [41]. This research work is incorporating a well-defined Kalman Filtering (KF) approach to reduce the measurement error of the respective scanner [42]. The standard KF equations have shown in Eqs (9) and (10) to predict the mean and related variance-co variance values.


$$X_{m}=AX_{n-1}\;+\;BU_{n}$$ (9)

$$P_{m}=AP_{n-1}A^{T}+\;Q$$ (10)

Here *X*_*m*_ and *P*_*m*_ are the predicted mean and covariance matrices, *X*_*n*−1_ and *P*_*n*−1_ are the last estimated mean and covariance matrices, *U*_*n*_ is the control vector along with *B* as its coefficient matrix, *A* is the system Jacobean matrix and *Q* is the process noise. In the calibration scheme of this work, each individual range measurement of the scanner has been estimated to get its respective mean value *X*_*n*_ in KF formulation. There is no control input involved in the sensing application and *A* becomes unity due to single variable prediction so Eqs 9 and 10 have reduced to *X*_*m*_ = *X*_*n*−1_ and *P*_*m*_ = *P*_*n*−1_ + *Q* respectively. In the correction phase of standard KF algorithm, the following equations from (11)–(13) have been used to determine the required KF parameters using the current measurement *z*_*n*_ and its respective noise *R* as shown below:

$$y=z_{n}-\;HX_{m}$$ (11)

$$S=HP_{m}H^{T}+\;R$$ (12)

$$K=P_{m}H^{T}S^{-1}$$ (13)

Here *y* is the innovation term, *S* is the covariance and *K* is the Kalman gain. The current range measurement *x*_*i*_ is used as *z*_*n*_ with *R* as the manufacturer’s provided variance value while *H*, the measurement Jacobean, is used as unity due to single variable estimation. So Eqs (11)–(13) have reduced to y = *x*_*i*_ − *X*_*m*_, *S* = *P*_*m*_ + *R* and *K* = *P*_*m*_*S*^−1^ respectively. Finally, the estimated mean range measurement *X*_*n*_ and its variance *P*_*n*_ have been determined by using the standard KF Eqs (14) and (15).


$$X_{n}=X_{m}+\;Ky$$ (14)

$$P_{n}=(I-KH)P_{m}$$ (15)

Here *X*_*n*_ is the new estimated mean range measurement and represents the term ${\overset{-}{x}}_{m}$ which was calculated with an algebraic formulation in earlier sections. While *P*_*n*_ is the variance estimate of the range variable and represents the similar term of ${{\overset{-}{\sigma }}_{m}}^{2}$ as determined earlier. The KF formulation from Eqs (9)–(15) has been processed continuously whenever a new range measurement *x*_*i*_ has been received and therefore new estimations of mean and variance have been iteratively generated. This mechanism has been applied individually on all scanners for the recorded test measurements as discussed in section 4.1. The plot of the estimated mean range values for the initial thousand samples has shown in Fig 24. The estimated mean range measurements of URG-04LX and UTM-30LX have appeared quite close to the true value while RPLidar has shown a relatively large shift from the true value. All the estimated mean values of scanners are showing stable responses with minute deviations if compared with the earlier results of mean values as shown in Figs 9–11. The estimated standard deviation has been significantly reduced to half of the value as compared to the manufacturer’s values provided in the datasheets. Therefore, the KF formulation has efficiently reduced the noises present in the range measurements and made it more stable and closed to the true values.

**Fig 24:** Plot of mean range measurements estimated through KF.

## 6. Conclusion

The comparative analysis of various compact and economical 2D laser scanners including Hokuyo URG-04LX, RPLidarA1 and Hokuyo-30LX is reported. These scanners were tested for possible usage in the backpack scanning and mapping system for indoor environments. During the tests, all the scanners exhibited fairly acceptable performance by working under the limits on various parameters as mentioned in the provided data sheets with minute exceptions of outliers. In order to further study their characteristics related to environmental and operational conditions, many tests have been conducted and presented in the paper. It is primarily observed that each scanner has a drift in range measurements due to heating effect of the scanner. The Hokuyo-04LX scanner has almost reached the acceptable range stability after twenty minutes of operation while the low cost RPLidar A1 scanner has shown a minute continuous change in the range values and never reaches to the stable measurements. The Hokuyo-30LX has emerged as the better scanner that reached acceptable stability within a few minutes of its working for short range applications and took approximately twenty minutes to reflect stability for medium range applications. It also exhibited consistency in standard deviations and in *RMSE* values irrespective of measuring range variations while the other two showed clear accumulation in both parameters especially RPLidar A1 has reflected broader deviations as measuring range increased. Due to low angular resolution, the Hokuyo-30LX has returned a greater number of points of any scanned object as compared to the other two scanners which is appeared it’s an additional advantage. In general majority of the materials which are commonly available in indoor environments such as wood, steel or concrete, have been tested through continuous scanning using all scanners and results have reflected almost similar behavior with minute deviations in the range measurements. However, the shiny vinyl plastic object has produced greater variations in the mean range, relative error and standard deviations for all scanners. In a similar manner, multiple scanning tests by changing the colors of targeted objects have been performed and nearly similar responses have been observed with minute variations in mean and standard deviations for all scanners. Therefore comprehensive testing of all scanners has provided a clear picture that the Hokoyu-30LX has the better performance capabilities in all technical parameters described in the paper and it has outclassed the others during multiple tests performed. However, its performance can be enjoyed only at a higher cost, which will certainly be a bottleneck for developing more economical systems at compromised performance. For this reason, Hokoyu-04LX has appeared a good choice for low range operations and showed quite stable and nearly accurate results as mentioned in the paper. Similarly, the RPLidar A1 has appeared comparatively less accurate scanner but it is available exceptionally at a low price, which makes it suitable for the economic system developments such as rover operations where it can provide a complete 2D slice of the surrounding region an affordable price. After completing the characterization of all scanners, a calibration scheme has been discussed to reduce the noises of scanners using the Kalman Filter mechanism. The developed results using the calibration scheme have found better than the earlier results observed without applying the calibration model. The noises in range measurements have clearly reduced to half of the previous values as depicted by the mean range and standard deviation parameters for all scanners as presented in the paper. Therefore, utilizing a calibration model with scanners is recommended in order to improve the measurement accuracy without consuming additional cost on hardware setups.

## Variables and constants

**Table:** 

$x_{i},\;{{\overset{-}{x}}_{m},\;\overset{-}{x}}_{M}$	Single range sample, sample mean, overall mean value for entire test	mm
$\sigma_{m},{\overset{-}{\sigma }}_{M}$	Standard deviation of samples, overall mean value of standard deviation for entire test	mm
$\eta_{m},{\overset{-}{\eta }}_{M}$	Relative error of samples, overall mean value of relative error for entire test	%
***RMSE***	Root mean square error	mm
***X***_***m***_, ***X***_***n***_	Predicted mean value, current estimated mean value	mm
***P***_***m***_, ***P***_***n***_	Predicted variance value, current estimated variance value	mm^2^
***R***, ***Q***	Constant measurement variance, constant process variance	mm^2^

## Acronyms

KF: Kalman Filter
ROS: Robot Operating System
SLAM: Simultaneous Localization And Mapping
